# Smart Healthcare System Based on Cloud-Internet of Things and Deep Learning

**DOI:** 10.1155/2021/4109102

**Published:** 2021-06-28

**Authors:** Benzhen Guo, Yanli Ma, Jingjing Yang, Zhihui Wang

**Affiliations:** College of Information Science and Engineering, Hebei North University, 11 Diamond South Road, Zhangjiakou 075000, China

## Abstract

**Introduction:**

Health monitoring and remote diagnosis can be realized through Smart Healthcare. In view of the existing problems such as simple measurement parameters of wearable devices, huge computing pressure of cloud servers, and lack of individualization of diagnosis, a novel Cloud-Internet of Things (C-IOT) framework for medical monitoring is put forward.

**Methods:**

Smart phones are adopted as gateway devices to achieve data standardization and preprocess to generate health gray-scale map uploaded to the cloud server. The cloud server realizes the business logic processing and uses the deep learning model to carry out the gray-scale map calculation of health parameters. A deep learning model based on the convolution neural network (CNN) is constructed, in which six volunteers are selected to participate in the experiment, and their health data are marked by private doctors to generate initial data set.

**Results:**

Experimental results show the feasibility of the proposed framework. The test data set is used to test the CNN model after training; the forecast accuracy is over 77.6%.

**Conclusion:**

The CNN model performs well in the recognition of health status. Collectively, this Smart Healthcare System is expected to assist doctors by improving the diagnosis of health status in clinical practice.

## 1. Introduction

By the end of 2015, there were about 220 million people aged 60 or above in China, accounting for 16.1% of the total population. Among them, 140 million were over 65 years old, accounting for 10.5% of the total population. In this context, healthcare for the elderly has increasingly aroused social concern [1]. The rapid development of wearable devices, IOT, and cloud computing has brought about significant development opportunities and affected every aspect of people's lives. In the field of healthcare, the adoption of IOT can bring us health monitoring all the time [2]. With the popularity of smart phones, smart bracelets, and other devices, a variety of sensors can monitor health indicators timely and accurately [3–5]. Deep learning is an implementation method of machine learning, which is different from the traditional shallow models such as artificial neural network. Deep learning usually has a deeper model structure with five or six layers or even over ten layers or more hidden layers [6]. In addition, the importance of feature learning is highlighted [7, 8]. The feature representation of samples in the original space is transformed into a new feature space by means of feature transformation layer by layer. Deep learning is widely used in image and voice processing and develops rapidly in the medical and health field [8–10]. The study in [11] proposed a human fall early warning algorithm based on RNN and compared it with traditional machine learning algorithms such as SVM to verify its excellent performance. The study in [12] compared and studied the application of CNN, RNN, LSTM, and other deep learning models in the evaluation of sleep quality.

With the increase of the number of IOT devices and sensors, medical IOT system also highlights more problems in the development process, mainly including the following:

1. The measurement parameters of existing wearable health monitoring devices are relatively simple, such as pedometers and intelligent sphygmomanometers. The common pedometer devices can connect with smart phones via Bluetooth and other communication means, and upload data to the cloud server, so it is possible to view data such as exercise amount and sports assessment report through the phone APPs. Various forms of wearable health monitoring devices fail to share data due to different manufacturers and communication protocols.
2. Limited by memory capacity and computing power, wearable devices may upload the collected data to the cloud server through smart phones or home gateways. The cloud server needs to store and process a large amount of collected data. The server and network have great transmission pressure, which reduces the real-time processing capacity.
3. At present, many telemedicine monitoring systems based on IOT carry out certain disease early warning according to a set of diagnostic schemes, and it is difficult to develop personalized diagnosis and treatment schemes according to individual physiological characteristics and historical parameter changes.
4. Intelligent diagnosis methods based on the uploaded data of health monitoring devices mainly include system-based diagnosis methods of experts and intelligent diagnosis methods based on sample data. Back Propagation (BP) neural network algorithm [13] and Support Vector Machines (SVM) algorithm have been applied to the classification of diagnosis results. Although deep learning algorithm has been applied in sleep quality and other fields [12], the application of intelligent diagnosis algorithm based on deep learning is rarely seen.

In view of the above problems, a healthcare monitoring system based on Cloud-Internet of Things (C-IOT) and deep learning is proposed, and the major work includes the following aspects:

1. A health data acquisition system is designed based on C-IOT and the acquisition of parameters such as human blood pressure, body temperature, body weight/fat, and exercise amount is realized. The shortcoming that the acquisition of simple physiological parameters fails to evaluate and diagnose the user's health effectively is avoided.
2. Data preprocessing of each acquisition device is realized locally to eliminate noise interference. By communicating with the user's smart phones through Bluetooth, the smart phones may display the collected data in real time, preprocess the data of each device, and upload them to the cloud server. The processing and integration of local data can reduce the computing pressure of cloud server and transmission pressure of network.
3. The private doctor evaluates the user's health condition according to the data on the cloud server and establishes the initial data set. The cloud server uses the deep learning algorithm (CNN) to train the user health evaluation model according to the initial data set. The newly uploaded data are calculated by a depth model to automatically give health assessment results. The model is a process of dynamic change. The private doctor will manually evaluate the user's health status and update the user data set on a regular basis as well as the parameter values of the depth model. The model can realize personalized health assessment.

## 2. Materials and Methods

### 2.1. System Architecture

Figure 1 indicates the architecture of health monitoring system based on C-IOT and deep learning proposed in this paper. It is improved from the traditional three-layer architecture of the IOT, and described from the perspective of system implementation and data flow, including data collection layer, data preprocessing and net layer, data processing, and application layer.

Data collection layer is responsible for the acquisition of physiological parameters of health, which is mainly composed of a number of Internet-connected or wearable devices. Temperature, body fat/weight, blood pressure parameters, and exercise parameters are measured. In general, data collection layer devices have small data storage capacity and low computing capacity [14–16]. In order to reduce data redundancy, network transmission pressure, and power consumption, the data denoising, digital filtering, and power management based on rules can be realized locally. High-frequency noise is eliminated by digital low-pass filter and band-pass filter. In addition, the special value in the collected data is removed based on rules. The data collection layer device may be connected to smart phones or other mobile intelligent terminals through Bluetooth.

The data preprocessing and net layer are mainly composed of smart phones and other intelligent mobile terminals. Smart phone devices not only serve as network layer devices to realize data communication function of medical IOT gateway, but also install application layer APP software to realize local data preprocessing, parameter display, and device control. The smart phone connects to the data collection layer device through Bluetooth to receive measurement information reported by the blood pressure meter, weight/fat meter, pedometer, thermometer, and other data acquisition devices, and display the real-time information on the mobile APPs. Preprocessing data are uploaded to the cloud server through Wifi, 4G, and other communication means. Data preprocessing includes data normalization, data dimension transformation, data fusion, and other functions to generate images of health parameters. In terms of data normalization, body weight, body temperature, and other measurement parameters are normalized according to the grade to the gray value ranging from 0 to 255. In terms of data dimension transformation, original measurement parameters are extended in dimension, such as heart rate, systolic pressure and diastolic blood pressure measured by sphygmomanometer extended to ambulatory pulse pressure (APP), mean arterial pressure (MAP), and ambulatory rate-pressure product (ARPP), which are often used to diagnose cardiovascular diseases more effectively. The application software of mobile phones can also fuse the physiological parameter measurement data after normalization of gray value and dimension expansion into the image of health parameters, upload them to the cloud server in the form of two-dimensional image, and use the deep learning model to solve the health parameter image to give the health index report. The users may receive and display the health report issued by the cloud server through smart phones. Making full use of the computing power of intelligent equipment for data preprocessing can effectively reduce the transmission pressure of database and network. With the rapid improvement of the computing power of intelligent terminal equipment, more and more data processing functions will be completed directly in the intelligent terminals.

The data processing and application layer mainly includes database and distributed server, web server, and deep learning model engine. The database stores and manages users' personal information/health monitoring data, personal doctor information, equipment information, etc., the distributed server realizes various business processing logic, and the web server provides users and personal doctors with friendly web interface for background operation. The deep learning model engine is used to train the deep learning model, and the trained deep learning model is used to solve the health parameter image. With the increase of user data, private doctors can annotate the data, enrich the personal health data set, and retrain and update the deep learning model.

### 2.2. Measurement of Blood Pressure

For blood pressure acquisition nodes, the oscillometric method is used to measure blood pressure [17], and the pressure value of the pressure sensor is filtered by low-pass filter and band-pass filter to obtain the static pressure value and the dynamic pressure value. In the measurement process, the dynamic pressure value amplitude increases gradually and then decreases. When the dynamic pressure value amplitude is multiplied by the normalized coefficients (*Ks* and *Kd*), the dynamic pressure value amplitude corresponding to the systolic pressure and the diastolic pressure can be obtained, respectively, and the human blood pressure value can be obtained by reverse check, as shown in Figure 2. According to the conclusions of Mauro's mathematical model, the normalized coefficient *Ks* was 0.46–0.64, and the normalized coefficient *Kd* was 0.43–0.73 [18]. In this paper, the amplitude coefficients commonly used in clinical medicine are *Ks* = 0.48 and *Kd* = 0.58 [19].

In order to obtain the optimal pulse oscillation amplitude envelope, Gaussian fitting method is used for data fitting: a set of sample data (*x*_*i*_, *y*_*i*_)(*i*=1,2,3 … *N*) can be described by Gaussian functions as shown in the following equation:

(1) $$\begin{array}{c} y_{i}=y_{\max}*\;\exp\left[-\frac{{\left(x_{i}-x_{\max}\right)}^{2}}{s}\right]. \end{array}$$

Take the logarithm of both sides of this equation:

(2) $$\begin{array}{c} \ln\;y_{i}=\ln\;y_{\max}-\frac{{\left(x_{i}-x_{\max}\right)}^{2}}{s}=\left(\ln\;y_{\max}-\frac{x_{\max}^{2}}{s}\right)+\frac{2x_{i}x_{\max}}{s}-\frac{x_{i}^{2}}{s}. \end{array}$$

Assume

(3) $$\begin{array}{c} \ln\;y_{i}=z_{i},\\ \ln\;y_{\max}-\frac{x_{\max}^{2}}{s}=b_{0},\\ \frac{2x_{\max}}{s}=b_{1},\\ -\frac{1}{s}=b_{2}. \end{array}$$

Taking all sample data into consideration, equation (2) is converted into a matrix as follows:

(4) $$\begin{array}{c} \left[\begin{array}{c} z_{1}\\ z_{2}\\ \vdots \\ z_{n} \end{array}\right]=\left[\begin{array}{ccc} 1 & x_{1} & x_{1}^{2}\\ 1 & x_{2} & x_{2}^{2}\\ \vdots & \vdots & \vdots \\ 1 & x_{n} & x_{n}^{2} \end{array}\right]\left[\begin{array}{c} b_{0}\\ b_{1}\\ b_{2} \end{array}\right]. \end{array}$$

It is simplified as

(5) $$\begin{array}{c} Z=XB. \end{array}$$

According to the principle of least squares, the generalized solution of least squares for matrix *B* is

(6) $$\begin{array}{c} B={\left(X^{T}X\right)}^{-1}X^{T}Z. \end{array}$$

Then, the estimated parameters (*b*_0_, *b*_1_, *b*_2_) are substituted into equation (1) to obtain the fitted Gaussian function. Both the measuring speed and accuracy are improved by using Gaussian fitting function.

### 2.3. Data Preprocessing

After the human physiological parameter monitoring equipment transmits the measurement results to a smart phone via Bluetooth, data preprocessing shall be conducted through the application software installed in the smart phone, which mainly includes dimensional transformation of data, data standardization, and generation of two-dimensional gray image for human health.

In order to optimize the input vector, the measurement data uploaded by monitoring equipment need to be transformed into a certain dimension. The measured data including heart rate (HR), systolic blood pressure (SP), and diastolic blood pressure (DP) are converted into three parameters, namely, mean arterial pressure (MAP), ambulatory pulse pressure (APP), and ambulatory rate-pressure product (ARPP).

(7) $$\begin{array}{c} \text{APP}=F1\left(\text{SP},\text{DP}\right)=\text{SP}-\text{DP},\\ \text{MAP}=F2\left(\text{SP},\text{DP}\right)=\frac{\text{DP}+\left(\text{SP}-\text{DP}\right)}{3},\\ \text{ARPP}=F3\left(\text{HR},\text{SP}\right)=\text{HR}*\text{SP}. \end{array}$$

Step number, motion distance, fast motion time, fast motion distance, length of sleeping, and length of awakening are obtained according to the step number and time measured by the pedometer after dimension expansion. Data standardization converts the data of each index into the gray value ranged from 0 to 255 according to the scaling, so as to facilitate the synthesis of health status matrix for uploading to the cloud server for processing. The corresponding range relationship between the measured value of each index and the standardized value is shown in Table 1.

In this paper, the deep learning method is adopted to evaluate the human health status. The input data of the deep learning model are the measured values after the standardization of each physiological parameter of human body in a day. In order to better serve as the input of CNN, the standardized data need to be processed in two dimensions to generate the health status matrix. The health status matrix is organized into 2D images. As required, the subjects shall have their blood pressure and body temperature measured once every morning and every evening, have their weight/fat measured once every day, and wear a pedometer 24 hours a day. On the smart phone side, 36-pixel 2D images of human health are generated every day, as shown in Table 2.  Figure 3 is an example 2D image of health status matrix according to Table 2.

### 2.4. Collection of Data Set

The training of deep learning model shall be supported by a certain amount of labeled data set. In this study, the gray-scale chart of health monitoring parameters in one day is obtained by combining measurement and construction. Six volunteers are selected, including 3 males and 3 females (including 2 adolescents, 2 middle-aged, and 2 elderly). The volunteers are required to test the blood pressure each morning and evening, the body temperature once, and the weight/fat once. They are also required to wear a pedometer device for 24 hours and upload data to the cloud server at 6 o'clock each morning through the phone APP. Then, private doctors will grade their health status according to the uploaded data and user information such as age and gender and then divide them into three types: health, sub-health, and illness. The initial data set is generated by continuously tracking and annotating the user's data for 100 days. In addition, the initial data set of each user constructed and annotated by private doctors according to the user's historical data information is 3,000, and these three types account for 1/3. 80% of the extended initial data set is selected as the training sample to train the user's personalized deep learning model, and 20% is used as the test sample to test the model's performance.

### 2.5. Deep Learning Model

Deep learning model is constructed and trained in the cloud server, and CNN is the most commonly used deep learning model, which has been widely used in the field of image processing. The classic LeNet-5 [20] CNN model is adopted and modified to simplify a pooling layer. The CNN model constructed is shown in Figure 4, which contains two convolution layers, a pooling layer, and a full connection layer. The CNNs have 2 × 2 kernels for the convolutional layers with 3 and 9 filters, respectively, and a scaling of 2 for the max-pooling layers. The output layer outputs the health assessment results, including health, sub-health, and illness.

## 3. Results and Discussion

### 3.1. Measurement and Test of Blood Pressure

The method of using medical blood pressure meter and blood pressure measurement node at the same time for the same subject is used for comparative verification. A health monitor (PM-900S, Biocare Technology Co. Ltd., Shenzhen, China) is selected as the comparison device. The verification results are shown in Table 3, and the measurement results indicate that the relative error is within the range of 6%.  Figure 5(a) is the photo of blood pressure measurement node device.

Also, the method of wearing commercial pedometer and step monitoring node is used for comparative verification. A sports bracelet (Honor 3, HUAWEI Technology Co. LTD, Shenzhen, China) is selected as the comparison experiment device. The test subjects wear sports bracelets and step monitoring nodes at the same time. The measured data of the previous day is read after the subjects get up at 6 o'clock in the morning. The verification results are shown in Table 4, and the measurement results indicate that the relative error is within the range of 9%.  Figure 5(b) is the photo of step monitoring node.

### 3.2. Evaluation of Deep Learning Algorithm and Model

For each subject, the accuracy of average recognition of the three health states is studied. Apart from that, recall and precision and *F*1_score are used for model evaluation in respect of each category [21]. The data of test set in data set are used as model input. TP denotes number of true positive (labeled correctly). FP denotes number of false positive (other activity labeled as the sub-health and illness). Furthermore, TN denotes number of true negatives (correct rejection), and FN denotes number of false negatives (missed detections).

(8) $$\begin{array}{c} \mathrm{Accuracy}=\frac{\mathrm{TP}+\mathrm{TN}}{\mathrm{TP}+\mathrm{FP}+\mathrm{FN}+\mathrm{TN}},\\ \mathrm{recall}=\frac{\mathrm{TP}}{\mathrm{TP}+\mathrm{FN}},\\ \mathrm{precision}=\frac{\mathrm{TP}}{\mathrm{TP}+\mathrm{FP}},\\ F1\_\mathrm{score}=\frac{2\mathrm{precision}*\mathrm{recall}}{\mathrm{precision}+\mathrm{recall}}. \end{array}$$

Figure 6 exhibits the accuracy of the average classification of each subject. Error bars display the standard deviation of the recognition accuracy of the three health categories for each subject. As can be seen from the figure, the results of different subjects are of obvious differences. The highest recognition accuracy of CNN model is 84.2% (S4) and the lowest is 68.5% (S3). The standard deviation of recognition accuracy is all within 15 and the maximum is 14.94 (S5). For 6 subjects, the average accuracy of CNN model is 77.61%.

Figure 7 indicates the confusion matrices of 6 subjects acquired by CNN model. It can be revealed that the recognition performance of the model for health categories is obviously superior to the other two categories. In 200 samples, the highest recognition accuracy is 182 (S6). The capability to recognize sub-health categories is relatively poor, and S5 can only recognize 110 out of 200 samples correctly.

Figure 8 shows the precision, recall, and *F*1-score of 6 subjects in three categories acquired by CNN model. It can be seen that CNN model boasts higher precision for disease recognition than other two categories, except S2. Nevertheless, the value of recall is higher than that of precision except S2. *F*1_score is a comprehensive index reflecting the performance of the model. By observing the *F*1_score curve of 6 subjects, the recognition performance of the model for sub-health is worse than the other two categories, with a minimum of 61.8% (S5).

The current research suggests that it is feasible to recognize and intelligently diagnose the preprocessed data of the underlying devices of the medical Internet of Things with CNN model. In comparison with traditional machine learning methods such as SVM [22] and LDA [23], the depth learning method for intelligent diagnosis does not require manual selection of data feature values. The depth model can automatically extract features and perform high-level abstraction. For different subjects, the optimal parameters of the model can be automatically acquired through training, which is more flexible and robust compared with traditional machine learning methods. The intelligent health management system architecture based on deep learning proposed in the current research can make the data set continuously grow under the condition of user data accumulation, and cooperate with doctors' manual annotation, and can optimize model training from time to time to achieve better recognition and diagnosis effects. Pretreatment of health data at the bottom layer of Internet of Things equipment enhances the robustness of data and can tremendously lower the computing pressure of servers.

For each subject, the accuracy of average recognition of the three health states is studied. Apart from that, recall and precision and *F*1_score are used for model evaluation in respect of each category.

## 4. Conclusions

In view of the existing problems in the existing IOT medical system, a new IOT architecture for medical monitoring is proposed in this paper, in which smart phones are used as gateway devices to realize data preprocessing of measurement node devices, thus greatly reducing the computing pressure of cloud servers and transmission pressure of network. Based on the data sets generated from such data annotated by private doctors, a CNN health recognition model is constructed to realize personalized diagnosis and treatment of human health. Six subjects are selected to wear wearable measuring devices for a long time and physiological parameters are measured as required. The test sample set is input into the deep learning model for identification, with a prediction accuracy of over 77%. In the future work, the measurement types of human health parameters will be added, such as ECG and EEG signals, etc. In addition, the scale of the data set will be expanded, and the training depth learning model will be updated continuously to improve the prediction accuracy.

## Figures and Tables

**Figure 1:** System architecture.

**Figure 2:** Blood pressure measurement method.

**Figure 3:** 2D images of human health.

**Figure 4:** CNN model architecture.

**Figure 5:** (a) Blood pressure measurement node device. (b) Step monitoring node device.

**Figure 6:** Classification accuracy of each subject. Each bar and the corresponding error bar show the average classification accuracy with standard deviation of three health patterns.

**Figure 7:** Confusion matrices acquired by the CNN model. (a–f) The confusion matrix of S1–S6.

**Figure 8:** Precision, recall, and *F*1-score obtained by the CNN model. (a–f) The result curves of S1–S6.

**Table 1:** Data standardization.

Index	Range of measurement value	Range of standard value
Weight	0–150 kg	0–255
Fat	0%–50%	0–255
SP	0–250 mmHg	0–255
DP	0–250 mmHg	0–255
HR	0–200 bpm	0–255
APP	0–200 mmHg	0–255
MAP	0–300 mmHg	0–255
ARPP	0–50000	0–255
Step num	0–30000	0–255
Distance	0–20 km	0–255
Fast motion time	0–24 h	0–255
Fast motion distance	0–20 km	0–255
Length of sleeping	0–24 h	0–255
Length of awakening	0–24 h	0–255
Body temperature	30–45°C	0–255

**Table 2:** Human health map.

	1	2	3	4	5	6

1	SP1	DP1	HR1	APP1	MAP1	ARPP1
2	SP2	DP2	HR2	APP2	MAP2	ARPP2
3	Weight			Fat		
4	Step num	Distance	Fast motion time	Fast motion distance	Length of sleeping	Length of awakening
5	Body temperature1					
6	Body temperature2					

**Table 3:** Blood pressure measurement verification results.

	SP (mmHg) (PM-900S)	SP (mmHg) (test node)	Error (%)	DP (mmHg) (PM-900S)	DP (mmHg) (test node)	Error (%)
1	120	123	2.5	83	86	3.6
2	107	112	4.7	78	82	5.1
3	124	130	4.8	89	86	3.4
4	109	105	3.7	78	81	3.8
5	140	145	3.6	95	99	4.2

**Table 4:** Step monitoring node verification results.

	Step num (honor3)	Step num (test node)	Error (%)	Amount of sleep (h) (honor3)	Amount of sleep (h) (test node)	Error (%)
1	5600	5743	2.6	6.5	6.3	3.1
2	8212	7920	3.6	7.4	7.0	5.4
3	15401	16280	5.7	8.2	7.7	6.1
4	7231	7102	1.8	7.1	6.6	7.0
5	11005	10098	8.2	9.4	9.0	4.3

## Data Availability

The data used to support the findings of this study are available from the corresponding author upon request.
